# Activation and selective IL-17 response of human Vγ9Vδ2 T lymphocytes by TLR-activated plasmacytoid dendritic cells

**DOI:** 10.18632/oncotarget.11755

**Published:** 2016-08-31

**Authors:** Elena Lo Presti, Nadia Caccamo, Valentina Orlando, Francesco Dieli, Serena Meraviglia

**Affiliations:** ^1^ Central Laboratory of Advanced Diagnosis and Biomedical Research (CLADIBIOR), University of Palermo, Palermo, Italy; ^2^ Department of Biopathology and Medical Biotechnologies (DIBIMED), University of Palermo, Palermo, Italy

**Keywords:** γδ T cells, plasmacytoid dendritic cells, IL-17, TLR activation, proliferation, Immunology and Microbiology Section, Immune response, Immunity

## Abstract

Vγ9Vδ2 T cells and plasmacytoid dendritic cells (pDCs) are two distinct cell types of innate immunity that participate in early phases of immune response. We investigated whether a close functional relationship exists between these two cell populations using an *in vitro* co-culture in a human system.

pDCs that had been activated by IL-3 and the TLR9 ligand CpG induced substantial activation of Vγ9Vδ2 T cells upon co-culture, which was cell-to-cell contact dependent, as demonstrated in transwell experiments, but that did not involve any of the costimulatory molecules potentially expressed by pDCs or Vγ9V2 T cells, such as ICOS-L, OX40 and CD40L. Activated pDCs selectively induced IL-17, but not IFN-γ, responses of Vγ9Vδ2T cells, which was dominant over the antigen-induced response, and this was associated with the expansion of memory (both central and effector memory) subsets of Vγ9Vδ2 T cells.

Overall, our results provide a further piece of information on the complex relationship between these two populations of cells with innate immunity features during inflammatory responses.

## INTRODUCTION

Plasmacytoid dendritic cells (pDCs) are one of the two principal subsets of human dendritic cells (DCs) and represent specialized cells for the production of type-I interferons (IFNs). They are involved in immune responses against most viruses and also act as a bridge between innate and adaptive immunity. pDCs comprise < 1% of total peripheral blood mononuclear cells (PBMCs) and can be isolated using antibodies against the surface markers BDCA-2 and BDCA-4. In humans, pDCs circulate in the blood of adults and neonates, can be located in lymphoid tissues, accumulate at inflammatory sites and also infiltrate various types of solid tumours. pDCs express a different profile of Toll like receptors (TLRs) than other subsets of DC, like TLR7 and TLR9, which are intracellular endosomal receptors for single stranded RNA and DNA [1–3]. Upon *in vitro* stimulation with interleukin (IL)-3 and TLR9 agonist-like CpG ODNs they acquire a typical DC morphology and many functional properties and participate to activation of other cell types like monocytes, B, NK and T lymphocytes.

Moreover, recent studies have shown that pDCs upregulate MHC class II molecules upon inflammation and induce both T cell mediated immunity and tolerance [4], thus highlighting their role in adaptive immunity.

Vγ9Vδ2 cells represent a major peripheral blood γδ T cell subset in humans (up to 1/20 of the peripheral blood lymphoid pool), which display broad reactivity against microbial agents and tumors. They recognize phosphoantigens (PAgs) of microbial (intermediates of the non-mevalonate (MVA) pathway of isoprenoid biosynthesis) and endogenous (metabolites of the MVA pathway) origin, whose production is upregulated upon cell stress [5]. Pharmacological agents can block either upstream (statins) or downstream (aminobisphosphonates (ABPs), alkylamines) MVA pathway leading, respectively, to decreased or increased intracellular isopentenyl pyrophosphate (IPP) levels. Alternatively, IPP could be presented by surface receptors unrelated to the MVA pathway. In fact, IPP metabolites can be converted into triphosphoric acid 1-adenosin-5′-yl ester 3-(3-methylbut3-enyl) ester (ApppI), an ATP analogue, which could then be processed and presented at the cell surface. Butyrophilin (BTN) 3A1 molecule controls activation of human Vγ9Vδ2 T cells by direct or indirect presentation of self and non self PAgs.

Similar to CD4 and CD8 T cells, Vγ9Vδ2 T lymphocytes are heterogeneous and comprise distinct populations that can be distinguished on the basis of surface marker expression and effector functions, such as cytokine secretion and cytotoxicity. Naive (T_naive_) CD45RA^+^CD27^+^ and central memory (T_CM_) CD45RA^−^CD27^+^ cells express lymph node homing receptors, abound in lymph nodes, and lack immediate effector functions. Conversely, effector memory (T_EM_) CD45RA^−^CD27^−^ and terminally differentiated (T_EMRA_) CD45RA^+^CD27^−^ cells express receptors for migration to inflamed tissues, are poorly represented in the lymph nodes while abounding at sites of inflammation, where they display immediate effector functions (cytokine production and cytotoxicity, respectively) [6].

Since γδ T cells and pDCs represent distinct components of the innate compartment, we investigated on their interactions and the underlying mechanism.

## RESULTS

### TLR-9 engagement on human pDCs induces Vγ9Vδ2 T cell proliferation

Previous studies have shown that Vγ9Vδ2 T cell clones secrete IFN-γ upon 24-hrs *in vitro* stimulation by TLR8/9-activated pDCs [7]. To ascertain the influence of pDCs on resting Vγ9Vδ2 T cells, immature pDCs or pDCs that had been activated by IL-3 and the TLR9 ligand CpG-A ODN2216, were cultured *in vitro* with CFSE-labelled Vγ9Vδ2 T cells freshly sorted from PBMC of healthy donors. Proliferation was assessed after 6 days of culture according to loss of CFSE labelling. Cumulative data from 12 individual experiments, expressed as the mean ± SD, are shown in Figure 1a, and representative data are shown in Figure 1b.

**Figure 1:** Human activated pDCs induce Vγ9Vδ2 T cells proliferation Immature or activated pDCs were co-cultured with purified, CFSE-labeled Vγ9Vδ2 T cells for 6 days. **a.** shows cumulative data of Vγ9Vδ2 T cells division, as assessed by CSFE. Error bars indicate the mean with SD (*p < 0.05) from 12 individual experiments, each carried out in triplicate. **b.** shows flow cytometry histogram of a representative experiment. Viable lymphocytes were gated by forward and side scatter, and analysis was performed on 100,000 acquired events for each sample by using FlowJo and the following gating strategy to detect lymphocytes: FSC/SSC, live cells, single cells, double positive CD3 and Vγ9Vδ2 T cells.

Immature pDCs induced significant Vγ9Vδ2 T cells proliferation (18.1% ± 2), but IL-3 and CpG-A activated pDCs induced substantial proliferation (48.3% ± 12.5) which was comparable to that achieved by Vγ9Vδ2 upon stimulation with the homeostatic cytokines IL-7 and IL-15 (60.3% ± 17) used as positive controls. Culture with IL-3 and CpG-A alone failed to induce detectable proliferation of Vγ9Vδ2 T cells (1.8% ± 1.1), thus excluding any direct effect of these two stimuli on Vγ9Vδ2 T cells.

Proliferation of Vγ9Vδ2 T cells was strictly dependent on the number of activated pDCs, with significant proliferation achieved at pDCs/Vγ9Vδ2 T cell ratio of 1:1 and 5:1, while no proliferation of Vγ9Vδ2 T cells was detected when the number of activated pDCs was lower than that of Vγ9Vδ2 T cells (0.1:1 and 0.01:1 ratios).

Figure 2a shows cumulative data from 5 individual experiments and Figure 2b shows representative data.

**Figure 2:** Enhanced proliferation of Vγ9Vδ2 T cells with higher pDC/V9Vδ2T cells ratio **a.** Percentage of proliferating Vγ9Vδ2 T cells at different pDC:Vγ9Vδ2 T cells ratio are shown. **b.** Flow cytometry panels (histogram plots) of a representative experiment are shown. The gating strategy is the same as described in the legend to Figure 1.

### pDCs-induced Vγ9Vδ2 T cell proliferation requires cell to cell contact

Vγ9Vδ2 T cells required contact with activated pDCs to proliferate, because when the cells were co-cultured separated by a transwell membrane to allow free exchange of soluble factors between upper and lower chambers in the absence of contact, Vγ9Vδ2 T cells consistently failed to proliferate (Figure 3a). To further exclude the possibility that pDCs-induced Vγ9Vδ2 T cell proliferation was due to soluble factors produced upon contact between these two populations, activated pDCs and Vγ9Vδ2 T cells were put together in the upper chamber and CFSE-labelled Vγ9Vδ2 T cells were cultured in the lower chamber. As shown in Figure 3a, Vγ9Vδ2 T cells failed to proliferate even under this experimental condition, clearly indicating that pDCs-induced proliferation of Vγ9Vδ2 T cells requires cell to cell contact and no soluble factor is involved in this interaction.

**Figure 3:** pDCs-induced Vγ9Vδ2 T cells proliferation requires cell to cell contact **a.** Frequency of proliferating Vγ9Vδ2 T cells when put in cell to cell contact, or in transwell experiment with or without contact (*p < 0.01). **b.** Vγ9Vδ2 T cell proliferation by pDCs in the presence of mAbs to CD40L, ICOS-L and OX40. Isotype-matched mAbs and medium alone were used as controls. Error bars indicate the mean ± SD (*p < 0.01). **c.** Flow cytometry panels of a representative experiment demonstrate the percentage of proliferating Vγ9Vδ2 T cells in presence of CD40L, ICOS-L and OX40 blocking mAbs, using the gating strategy described in the legend to Figure 1.

In previously published papers, different membrane molecules have been implicated in Vγ9Vδ2 T cell activation induced by several cell types including myeloid DCs, monocytes and NK cells [8]. Hence, a large panel of molecules potentially expressed by pDCs or Vγ9Vδ2 T cells, including the γδ TCR, CD3, NKG2D, CD80, CD86, CD40L, ICOS-L, OX40, and CD11, was screened using specific mAbs. However in our experimental model, blocking of any individual costimulatory molecule did not affect proliferation of Vγ9Vδ2 T cells (data not shown). mAbs to ICOS-L and CD40L caused an approximately 30% inhibition of pDCa-induced Vγ9Vδ2 T cell proliferation (Figures 3b and 3c), but inhibition did not attain statistical significance and did not increase upon addition of the two mAbs together (data not shown). Altogether, these results indicate that Vγ9Vδ2 T cell proliferation by pDCs does not require any of the tested membrane-bound costimulatory molecules. Thus, although interaction between cell surface molecules and counter ligands is involved, the nature of these molecules remains unclear at the moment.

### pDC-expanded Vγ9Vδ2 T cells show central memory phenotype

In order to assess the differentiation pattern of pDC-expanded Vγ9Vδ2 T cells, staining for CD45RA and CD27 was performed on Vγ9Vδ2 T cells after 6 days of co-culture with activated pDCs (Figures 4a and 4b) [9]. As expected, the majority of Vγ9Vδ2 T cells purified from buffy-coats had a T_CM_ phenotype (60% ± 5), but also consisted of cells with a T_EM_ phenotype (24.8% ± 5) and few cells with T_naïve_ (14% ± 4) and T_EMRA_ (0.7% ± 1) phenotypes.

**Figure 4:** pDCs-expanded Vγ9Vδ2 T cells have memory phenotype Vγ9Vδ2 T cells were cultured with pDCs or other stimuli as described in Materials and Methods. At the end of the culture period, cells were stained with mAbs to CD45RA and CD27 after gating on the Vγ9Vδ2^+^ T cells population. **a.** Bar graphs (mean ± SD) and **b.** flow cytometry analysis of one representative experiment.

After culture with activated pDCs, the majority of cells retained T_CM_ (50% ± 7) and T_EM_ (35% ± 7) phenotypes, while the percentage of naive cells decreased (from 14% ± 4 to 10% ± 2).

PAg (BrHPP)-activated Vγ9Vδ2 T cells showed a predominance of T_EM_ (54% ± 3) and T_CM_ (42% ± 9) phenotype, while Vγ9Vδ2T cells that had been stimulated with BrHPP and activated pDC showed a similar phenotype distribution to those cultured with pDCs alone. These results indicate that activated pDCs trigger Vγ9Vδ2 T cell division with maintenance of a T_CM_ phenotype, but are poorly capable to promote long-term *ex vivo* differentiation of activated Vγ9Vδ2 T cells into effector memory cells.

### Activated pDCs selectively induce IL-17 production by Vγ9Vδ2 T cells

We next analysed if activated pDCs could induce cytokine production by Vγ9Vδ2 T cells. Responses were compared to those promoted by the Vγ9Vδ2 T cell-specific PAg BrHPP, which is well known to trigger a range of type-1 cytokines production (IFN-γ and TNF-α) by Vγ9Vδ2 T cell lines. Intracellular FACS analysis (Figures 5a and 5b) showed that activated pDCs induced very poor, if any, IFN-γ production by Vγ9Vδ2 T cells, as compared to stimulation by Ionomycin and PMA used as a positive control (4.43% ± 0.23 *versus* 40% ± 2). BrHPP activated Vγ9Vδ2 T cells also produced significant IFN-γ (11.8% ± 3). Surprisingly, we found that Vγ9Vδ2 T cells were allowed to produce significant amounts of IL-17 upon co-culture with activated pDCs, while none of the other tested stimuli was capable to induce IL-17 production. Similar results were obtained by the measurement of IL-17 and IFN-γ concentrations in culture supernatants by ELISA (Figure 5c).

**Figure 5:** pDCs-expanded Vγ9Vδ2 T cells preferentially produce IL-17 **a.** Cumulative data of IFN-γ and IL-17 producing Vγ9Vδ2 T cells in the presence or absence of activated pDCs or other stimuli. Data shown are mean ± SD. **b.** shows flow cytometry panels of a representative experiment. **c.** ELISA of IL-17 and IFN-γ in supernatants of Vγ9Vδ2 T cells cultured for 6 days with pDCs or other stimuli. Data are shown as mean ± SD and are representative of three separate experiments, each carried out in triplicate.

## DISCUSSION

It is generally accepted that T cell differentiation, expansion and survival are enforced in response to cues delivered by DCs. In humans, DCs are divided into two classes: myeloid and plasmacytoid DCs [10, 11]. These latter are a unique population of bone-marrow-derived immune cells that reside primarily in lymphoid organs in the steady state, entering the lymph nodes from the blood [12, 13]. pDCs express endosomal nucleic acid-sensing TLR7 and TLR9 and respond to the respective ligands. The most distinct pDC response to these stimuli is rapid and abundant type-I IFN secretion [14]. Other consequences of TLR-induced pDC activation include the secretion of cytokines such as TNF-α and (in the mouse) IL-12 and the acquisition of antigen presentation ability. In addition to cytokine secretion, activated pDCs undergo a characteristic DC maturation program involving upregulation of co-stimulatory molecules and acquisition of T cell stimulation capacity. Altogether, these powerful immunostimulatory functions of pDCs contribute to the recruitment and/or activation of nearly all immune cell types [15, 16], establishing pDCs as a key link between innate and adaptive immunity.

A previously published study has shown that Vγ9Vδ2 T cell clones secrete IFN-γ upon 24-hrs *in vitro* stimulation by TLR8/9-activated pDCs [7], but it is still unclear whether pDCs cells can induce full activation of resting Vγ9Vδ2 T cells upon TLR ligand stimulation.

In this study we show that pDCs activated by TLR stimuli and IL-3 are fully capable to induce proliferation of Vγ9Vδ2 T cells at a 1:1 or 5:1 pDC/Vγ9Vδ2 T cell ratio.

Previous reports have demonstrated efficient *in vitro* DC maturation mediated by PAg- or aminobisphosphonate-stimulated Vγ9Vδ2 T cells [17], which involved both membrane-bound (i.e. CD40L) and soluble (i.e. TNF-α and IFN-γ) T cell-derived signals [18]. In our experimental model, transwell experiments clearly demonstrated that pDCs-induced proliferation of Vγ9Vδ2 T cells primarily involves cell to cell contact and does not require soluble factors. The possible implication of several candidate costimulatory molecules differentially expressed by pDCs was studied by means of blocking reagents, but did not led to any conclusive results to date. Analysis of the effect of inhibitors of various signalling cascades as well as transcriptome analysis of maturing pDCs at various time points should certainly help to identify the mechanisms underlying such a potentiation effect. In addition, given that ICOS and OX40 are involved in the tolerogenic properties of pDCs [19, 20], we performed blocking studies using anti-OX40, anti-CD40L and anti-ICOSL, all of which failed to inhibit pDCs-induced Vγ9Vδ2 T cells proliferation.

Surprisingly, and in contrast with previously published findings, activated pDCs selectively induced IL-17 responses of Vγ9Vδ2T cells, and this was associated to the expansion of memory (both central and effector memory) subsets of Vγ9Vδ2 T cells. In fact, a previous study showed that pDCs stimulated by CpG ODN2216 induced exclusive IFN-γ production by Vγ9Vδ2T cell clones in a 24 hrs co-culture. This was attributed exclusively to type-I IFN produced by TLR-stimulated pDCs. In agreement with data here reported, in rats and mice mature pDCs, but not myeloid DCs, support Th17 differentiation from naive T cells through secretion of high amounts of IL-6 [21]. Similarly, human peripheral blood-derived pDCs activated with IL-3 and CpG secrete high amounts of IL-6 and TNF-α, in addition to type-I IFN, but fail to promote IFN-γ production upon co-culture with naive CD4 T cells [22]. Moreover, human and mouse pDCs promote differentiation of Th17 responses upon TLR-mediated activation [23, 24]. Finally, pDCs efficiently induced the differentiation of T cells producing only IL-22 (Th22) in naive T cells, in an IL-6- and TNF-α-dependent way [25]. Altogether, these results underline that pDCs have an intrinsic unique capacity to induce IL-17 and or IL-22, but not IFN-γ secretion from T cells, including Vγ9Vδ2 T cells.

Typically, human Vγ9Vδ2 T cells default toward type 1 cytokine production and predominantly produce IFN-γ upon activation. However, under appropriate culture conditions, Vγ9Vδ2T cells divert from this typical Th1-like phenotype and polarize to different cytokine-producing subsets. Thus, the addition of IL-1β, IL-6, IL-23, and TGF-β in combination with TCR triggering promotes expression of the transcription factor RORC and polarization to IL-17-producing Vγ9Vδ2 T cells, while stimulation by cytokines alone did not enhance IL-17 production. This finding is consistent with the idea that Vγ9Vδ2 T cells are polarized T cells and the cytokine milieu can further drive their differentiation. The commitment and plasticity of effector T cell subsets are probably regulated by the expression and balance of lineage-specifying transcription factors, antigenic stimulation, or cytokine microenvironment, suggesting that Vγ9Vδ2 T cells may differentiate into multifunctional cells able to trigger additional responses in the periphery [27].

Previous studies have demonstrated that murine γδ T cells are an innate source of IL-17 without the need for TCR engagement by antigen [28–30]. A striking consequence of these findings is that the role of the TCR in IL-17-producing γδ T cells could be redundant, in line with their predetermined phenotype in the thymus without positive or negative selection. Accordingly, murine γ T cells acquire IL-17-producing potential in the neonatal thymus independently on encountering the specific antigen.

In contrast to mouse studies, TCR engagement is required for the differentiation of human IL-17-producing Vγ9Vδ2 T cells from naive precursors, which poses the question of how Vγ9Vδ2 T cells are stimulated to produce IL-17 by activated pDCs, apparently in the absence of TCR engagement.

In accordance with our results, Guery et al. [31] have demonstrated that Ag-presenting activated pDCs induce potent antigen-specific Th17 cells, suggesting that pDCs could be used not only as inflammatory cytokines producers but also as efficient APCs to improve tumor vaccine efficacy. Moreover, Takagi et al. [32] showed that in a murine model pDCs contribute to the generation of IL-17 producing γδ T cells under TLR7-mediated inflammatory conditions, that play a crucial role in the initiation of psoriasiform plaque formation [33–34].

In conclusion, our results demonstrate for the first time that TLR-activated human pDCs stimulate proliferation and promote selective IL-17 responses of Vγ9Vδ2 T cells in an innate fashion, thus providing a mechanism through which these two populations of cells with innate immunity features may interact at sites of inflammation.

## MATERIALS AND METHODS

### Human subjects

Peripheral blood mononuclear cells (PBMC) were isolated from buffy-coats of healthy donors, obtained from the Blood Bank of the University Hospital “P. Giaccone”, Palermo. All participants wrote informed consent.

### pDC and Vγ9Vδ2 T cells purification

PBMCs were obtained by density gradient sedimentation using Ficoll/Hipaque (Pharmacia Biotech, Uppsala, Sweden). To isolate pDCs, PBMCs were pre-enriched using anti-BDCA-4 PE mAb and anti-PE microbeads (MACS; Miltenyi Biotec, Bergisch Gladbach, Germany), according to the manufacturer's instructions, and sorted by using a FACS Aria Cell Sorter (BD Biosciences, Mountain View, CA), which resulted in 99% purity. The cells were then resuspended in RPMI 1640 (Euroclone, UK) supplemented with 10% FCS (Hyclone, Invitrogen, Italy), L-glutamine (2 mM), Hepes buffer (10 mM), and gentamycin (10 μg/ml) (Sigma-Aldrich, Germany). pDCs were activated following culture for 24 hrs in the presence of interleukin-3 (IL-3, R&D System, 10μg/ml) and CpGA-ODN 2216 (TIB MolBiol, 3 μg/ml) in 96-well flat bottom plates (Costar). γδ T cells were separated from PBMC by positive selection using anti-γδ-magnetic beads (Miltenyi Biotec) according to the manufacturer's instructions. Purified cell populations contained more than 98% of viable Vγ9Vδ2 T cells as assessed by flow cytometry.

### Co-colture of Vγ9Vδ2 T cells and pDC

Vγ9Vδ2 T cells were labelled with CFSE (Molecular Probes, Eugene, USA) and 2×10^5^ Vγ9Vδ2 T cells were co-cultured with 2×10^5^ activated pDC, in 96-well round bottom plates (Costar, Cambridge, MA) for 6 days at 37°C, 5% CO_2_. As a control CFSE-labelled Vγ9Vδ2 T cells were cultured with the PAg bromohydrin pyrophosphate (BrHPP, a generous gift of Dr. Jean Jacques Fourniè, 10nM final concentration) and IL-2 (20 U/ml final concentration) as reported in Dieli et al [35]. IFN-γ and IL-17 levels were measured in 6-day culture supernatants by ELISA according to the manufacturer's instructions (R&D Systems). In some experiments, co-cultures were carried out in the presence of blocking mAbs to CD40L, ICOS-L and OX40 or isotype-matched mAbs (all purchased from BD Bioscience, and used at 10 μg/ml final concentrations). To study the cell contact requirement, Vγ9Vδ2 T lymphocytes were physically separated from pDCs by a semipermeable membrane using transwell plates (6.5-mm diameter, 0.4-μm pore size, Corning Glass Work, Corning, NY). Vγ9Vδ2 T cells on the lowest well were harvested after 6 days at 37°C by gentle pipetting in PBS, washed, resuspended in medium and used for further analysis.

### Flow cytometry analysis

The following antibodies were used: anti-IFN-γ, anti-IL17A, anti-CD3, anti-CD27, anti-CD45RA and isotype-matched control mAbs, labelled with different fluorochromes, all purchased from BD Bioscience, and used according to the manufacturer's recommendations. Vγ9Vδ2 T cell proliferation was assessed after 6 days of co-culture according to loss of CFSE labelling in PI^−^ cells. To study intracellular IFN-γ and IL-17, Vγ9Vδ2 T cells were co-cultured with activated pDCs, Ionomycin and PMA or with BrHPP in the presence of monensin for the last 5 hrs at 37°C in 5% CO_2_. The cells were harvested, washed twice in PBS with 1% FCS and fixed with PBS containing 4% paraformaldehyde overnight at 4°C. Fixation was followed by permeabilization with PBS containing 1% FCS, 0.3% saponin, and 0.1% Na azide for 15 min at 4°C. Staining of intracellular cytokines were performed by incubation of fixed permeabilized cells with FITC-labelled anti-IFN-γ and APC-labelled anti-IL17A mAbs. After two more washes in PBS containing 1% FCS, the cells were analyzed by FACS CANTO II flow cytometer (BD Bioscience). Viable lymphocytes were gated by forward and side scatter, and analysis was performed on 100,000 acquired events for each sample by using FlowJo and the following gating strategy to detect lymphocytes from FSC/SSC, live cells, single cells, double positive CD3, and TCR Vγ9Vδ2 cells.

### Statistical analysis

Data were analyzed with Mann-Whitney test, and two-tailed Student's t test was used to compare significance of differences between groups. Data from different experiments were compared using one-way ANOVA Kruskal-Wallis multiple comparison test with Bonferroni correction, by usingGraphPad. Values of *p* < 0.05 were considered statistically significant.
